# Identification Model of Writhing Posture of Classical Dance Based on Motion Capture Technology and Few-Shot Learning

**DOI:** 10.1155/2022/8239905

**Published:** 2022-05-10

**Authors:** Ning Zhang

**Affiliations:** Shandong University of Arts, Jinan 250000, China

## Abstract

Chinese classical dance is cut into the inner verve from a grasp of external form in dance instruction, and the aesthetic fashion and artistic norms of classical dance are established with historical depth. The “professional specificity” of characters and the “language description” of plots are eliminated in Chinese classical dance creation, highlighting the contemporary spirit of classical dance creation. Chinese classical dance was born during the early years of the People's Republic of China. The term “classical dance” did not refer to all Chinese classical dances at the time; rather, it referred to a dance form that embodied China's national spirit and had a classical cultural heritage based on Chinese traditional dance. The average frequency of step-over was 0.9, which was higher than the average rate of basic turnover of 0.75 and step-by-step turnover of 0.5, according to the results of the SPSS19.0 analysis. As a result, except for a few points with loud noise, it can be concluded that stepping over is an effective feature. The recognition model of the somersault posture of classical dance is studied in this paper, a database for real-time acquisition of three-dimensional data of human motion is established, and the Google model of human body characteristics is obtained based on feature plane matching of human body posture, all using motion capture technology and few-shot learning. The above data has good reference and application value for improving teachers' teaching level and arousing students' learning enthusiasm in the dance teaching process when applied to posture teaching and analysis. The captured data can convert human motion in real three-dimensional space into data in virtual three-dimensional space. Motion capture technology converts human motion information into a technology that can be recognized by computers.

## 1. Introduction

Chinese classical dance is made up of traditional Chinese opera, dance, martial arts, and ancient art resources that are mined, screened, and integrated. “Twist, tilt, circle, curve, form, spirit, strength, and law” are the overall requirements and prominent features of Chinese classical dance, and these eight words evolve into posture and movement law through waist movement [1]. Second, in dance creation, Chinese classical dance should be cut from the understanding of external form to the understanding of internal charm, and the aesthetic fashion and artistic norms of classical dance have been established with historical depth; third, in dance teaching, Chinese classical dance should be cut from the understanding of external form to the understanding of internal charm, and the aesthetic fashion and artistic norms of classical dance have been established with historical depth; and fourth, in dance creation [2, 3], Chinese classical dance should be cut from the “profession specificity” of character images and the “ Opera,” which contains the living fossil of dance inheritance, was studied and learned by the founders of Chinese classical dance. The development of opera is perhaps a tributary in the great Chinese culture, but it is the most clear and complete [4]. The origins of Chinese classical dance can be traced back to the early days of the People's Republic of China. At the time, the term “classical dance” did not refer to all Chinese classical dances; rather, it referred to a dance form that embodied China's national spirit and had a classical cultural heritage based on Chinese traditional dance. When we consider that history, we cannot help but think of Mr. Ouyang Yuqian. He actively advocated for dancers learning the fundamental skills of Chinese opera, as well as studying and distinguishing Chinese classical dance from basic opera dance, and this suggestion was taken into consideration and implemented in the curriculum of the first dance school in New China [5, 6].

Motion capture system can track, monitor, and record human motion data. At present, it has been preliminarily applied and developed in entertainment effectiveness, health record, rehabilitation training, and other aspects [7, 8]. Motion capture is a process of acquiring the size measurement, position, and direction information of moving objects so as to realize further research. Since the 1970s, motion capture has been an important method of photographic image analysis in biomechanics research, and since then, this technology has been more and more widely used in animation, robot control, human-computer interactive games, sports training, and other fields [9]. The motion capture system is mainly composed of sensors, signal acquisition equipment, data transmission, and data processing, including mechanical, electromagnetic, and optical. The adopted motion capture equipment is an optical motion capture system with high precision and good stability, which has achieved ideal results in the process of collecting Xinjiang Uygur dance data [10, 11]. The dance data collected by the motion capture system is input into the 3D animation software and can be displayed perfectly through the virtual display engine [12]. Motion capture technology is a rapidly developed technology in the last 20 or 30 years. Many domestic and foreign researchers have invested a lot of scientific research efforts in this field and obtained advanced scientific research results and rich theoretical support in many aspects, including the way and application of motion capture, the analysis of real-time motion data, and the analysis of motion posture.

This paper proposes to apply the motion capture technology to the tumbling posture recognition model of classical dance, establish a database to obtain the three-dimensional data of human motion in real time, and match the human posture based on the feature plane to obtain the Google model of human characteristics. Applying the above data to the posture teaching and analysis in the process of dance teaching is helpful to improve the teaching level of teachers, Mobilizing students' learning enthusiasm has good reference and application value [13, 14]. Human motion posture analysis first rose abroad. With the advent of the new century, Chinese domestic research experts also began the research and analysis of three-dimensional posture [15].

This paper studies and innovates the above problems from the following aspects:

1. A writhing gesture recognition model of classical dance based on motion capture technology is proposed. This paper studies the identification model construction of the tumbling posture of classical dance. The combination of motion capture technology and the tumbling posture of classical dance will make up for the deficiency of traditional dance forms and has advantages that traditional dance does not have in the acquisition and transmission of movement skills. According to one's own state, one can study and demonstrate actions purposefully and then compare the analysis results of 3D motion data with the standardized action posture so as to correct the standardization of actions in time, which greatly improves students' learning and teachers' teaching efficiency.
2. Build the database of the identification model of the tumbling posture of classical dance based on motion capture technology. Based on the application of motion capture technology to the identification of the tumbling posture content of classical dance, firstly, set the performer's dance movements and their range of motion; then, capture the three-dimensional data of the performer's dance movements and establish a three-dimensional dance teaching model database. Finally, make the dance movement database into a three-dimensional animation and apply it to the identification model of the tumbling posture of classical dance.

The paper is divided into five parts, and the organizational structure is as follows:

The first chapter introduces the research background and present situation of the tumbling posture of classical dance and puts forward and summarizes the main tasks of this paper. The second chapter introduces the domestic and foreign related work of the somersault posture of classical dance. The third chapter introduces the principle and model of motion capture technology. In chapter 4, the realization of the recognition model of tumbling posture of classical dance based on motion capture technology is introduced, and the performance of the model is compared through experiments. The fifth chapter is the full text summary.

## 2. Related Work

### 2.1. Research Status at Home and Abroad

Gaglio et al. proposed that the first trouble for Chinese classical dance to recognize the posture from opera is the contradiction between “stylized dance and functional training,” which is the basic contradiction in the construction of Chinese classical dance teaching materials, which has not been completely solved until today [16]. TNA B proposed that the formation of “form” of Chinese classical dance was fundamentally influenced by ancient traditional concepts, mainly the concept of nature, and human natural activities affected the formation of artistic aesthetics and aesthetic ideas [17]. Shiqi et al. proposed that Mr. Mei Lanfang, an opera performing artist, is known as a male actress. When limited by certain clothing, props, and roles, how to shape the stage image of women's posture through a beautiful, “exquisite,” delicate, and “language” orchid palm has become an art form integrating the song, dance, and music of the previous generation [18]. Nai et al. proposed that classical dance comes from the burst of emotion, and Oriental people have formed a unique way of posture expression under the influence of traditional ideas. Easterners are not used to expressing their feelings directly like the West, but in a gentle and implicit way, which stems from the naive, simple, and restrained emotional thinking of farmers in the bones of Easterners [19]. The authors proposed that Chinese classical dance is a genuine domestic product and a new kind of dance comparable to modern dance and ballet. Most of its soundtrack is played with musical instruments with Chinese characteristics, such as pipa, erhu, guzheng, and Xiao, and the clothing usually has a smell of ancient fragrance [20]. Deng et al. proposed that the historical and cultural spirit precipitated in opera and dance is in the same line with the spirit of China's 5000-year-old traditional culture. We absorbed the orchid palm from it and drew lessons from and cited the “nonphysical performance” in the drama dance performance, which uses hand movements and human body posture with eyes, body method, pace, and so on [21]. Pope et al. put forward that the traditional poetry contains the ancient people's aesthetic thought activities in the aspects of appreciation and creation, which has a certain influence on the formation and development of Chinese classical dance [22]. Maheu et al. proposed to stand on the vision of the discipline construction of Chinese classical dance. The original intention of the course construction of body rhyme is to deepen the national attributes of Chinese classical dance styles, but it is still the historical mission of the discipline to cultivate the actors' body posture, and it is also an important project for the discipline to continuously inherit and spread the faculty with cultural heritage and professionalism [23]. Christopher et al. put forward that “the basic ability training of Chinese classical dance refers to the basic ability training and special quality training of all parts of body posture.” The basic skills training of Chinese classical dance mainly focuses on three aspects: strengthening the training of softness, training of quality and ability, and training of technical skills. From the ground, the lever, and the middle three parts, the soft opening strength of students and their technical skills can be solved [24]. Xuan et al. put forward that the body rhyme of Chinese classical dance should not only have the style of Chinese traditional body culture, but also conform to the scientific nature of human posture. Therefore, for the study of body rhyme of Chinese classical dance, discussing the principle of body rhyme capacity, the principle of style, and its practical application can provide important reference for the discipline to consolidate and deepen the theoretical foundation [25].

### 2.2. Research Status of Tumbling Posture Recognition in Classical Dance Based on Motion Capture Technology

This paper investigates the recognition of classical dance tumbling postures using motion capture technology. This paper examines the origin and transmission mechanism of the body rhyme movement power of Chinese classical dance from the perspective of human movement, in conjunction with traditional Chinese Dantian theory and the core of modern human physiological anatomy. This paper examines the principles of body rhyme movement in Chinese classical dance in terms of local form, overall movement law, and philosophical category from the standpoint of style; it then moves on to the application stage of action principle, which includes the application of principle in classroom teaching and the application of principle on stage. Human posture recognition and capture technology is currently the most widely used. The method for implementing it is to place the camera in a fixed position in space and then capture the object's real-time action and posture using light spots in this area. Classical art charm meets the rhythmic essence of traditional Chinese dance in China's classical dance. We must first determine the recognition target of human posture and the corresponding data acquisition scheme before recognizing the tumbling posture of classical dance. The main principle of attitude recognition and capture technology is to attach inertial sensors to the joints, such as a gyroscope and an accelerometer, to collect human attitude and action data, and then use data analysis and calculation to determine the amplitude and angle of human joint motion. The following are some of the advantages of this method: low price; there are no issues with the environment, such as light shielding, and the precision is excellent. This paper examines the significance of combining motion capture technology and dance teaching and verifies through experiments that using capture technology in teaching can improve students' subject status, as well as bring enlightenment and innovation to contemporary teaching research.

## 3. Principle and Model of Motion Capture Technology

The motion capture system records the movement process of moving targets using tracking devices with special marks placed at key positions. After that, computer processing is used to obtain three-dimensional space parameters, and finally, the matching of skeleton models used in animation is completed. The motion capture sensor's human behavior recognition technology is a multidisciplinary system that combines sensor technology, human dynamics, computer graphics, pattern recognition, and other disciplines. Front-end hardware and back-end software make up the technology. The front-end hardware's main functions and contents include gathering human motion data using motion capture sensors and transmitting that data to the computer. The back-end software's main purpose and content is to use the computer to efficiently process the collected exercise data so that the computer can automatically identify the action category of the captured object, allowing for action reproduction and human-computer interaction. First and foremost, the dancers' dance movements and range of motion should be established. The dance pose flowchart of the action capture technology of instructional design is shown in Figure 1.

While watching the animation, they draw posture movements in their mind. The actions that they do not understand or do not know can be demonstrated repeatedly from multiple angles. Secondly, students conduct practical demonstration, capture their own actions with high-precision three-dimensional camera, and compare them with teachers' standard actions. By comparing the dance movements with the teacher's standard movements in sections through the motion capture system, the shortcomings can be quickly found out, which is convenient for local correction. Motion capture technology is used to assist the teaching and research of dance. The early motion capture was proposed by American Polish Fisher in 1915. His “rotoscope” technology is considered to be the pioneer of motion capture technology. The main principle of this technology is to initially take the action video image taken in reality as the bottom sample of animation depiction, and then the animators depict the required actions frame by frame on this basis. The virtual display platform collects all kinds of dance materials, performs by actors, collects data through motion capture devices, and converts them into data recognizable by 3D animation software, and finally displays the dance content perfectly through the virtual display engine. The motion capture technology is applied to the data acquisition in the tumbling posture process of classical dance, the skeleton motion route of human body is extracted, and then the posture discrimination is obtained by using the feature vector matching method so as to establish the tumbling posture model of classical dance. It is easy to know that the depth of the whole bone tree is 3. The human body can be roughly divided into 11 bone trees, as shown in Figure 2.

The matrix algorithm is proved to be a feasible BVH analytical algorithm, as shown in formula (1), on how to convert the correct position and dynamic of bones into animation.

(1) $$\begin{array}{c} v{\;}^{\prime }=Mv. \end{array}$$

Type *v* indicates said transformation point; *v* indicates the original point; and *M* indicates the transformation matrix.

This formula is especially important when the matrix multiplication is three independent Euler angles, which are not exchangeable to construct the rotation matrix. Rotation matrix *R* is based on the rotation parameters of each axis of the individual rotation matrix, *R*_*x*_, *R*_*y*_, *R*_*z*_, as shown in formula (2), where the composition order is “*XYZ*.”

(2) $$\begin{array}{c} R=R_{x}R_{y}R_{z}, \end{array}$$

where *R* is rotation matrix; *R*_*x*_*y*is*y*-axis rotation parameter; *R*_*y*_*z*is*z*-axis rotation parameter; and *R*_*z*_*x*is*x*-axis rotation parameter.

The movement of a single bone consists of translation, rotation, and proportional components, which can be combined together and transformed by using homogeneous coordinates. Unless otherwise stated, the order of combination of these different transformations is stated in the form that sufficient transformations will always follow, such as the following formula.

(3) $$\begin{array}{c} M=TRS. \end{array}$$

Type *S* is said bone size and *T* is translation matrix.

In most motion capture file formats, the data is derived in a hierarchical way and formula, and formula (3) only gives the local transformation of a certain bone. The local transformation of the skeleton describes its direction in the local coordinate system, which in turn is influenced by the direction of its parent skeleton. Formula (4) lists this combination sequence, in which *n* − 1 is the current bone, its mother bone is *n*=0, and EE represents the root bone of the bone hierarchy.

(4) $$\begin{array}{c} M_{\text{global}}^{n}=\prod_{i=0}^{n}M_{\text{local}}^{i}. \end{array}$$

Using formula (4) and the derivation of local transformation, we can calculate the global position of the origin of each bone and obtain the position of the bone of the origin from the offset information of the hierarchy.

The function interval changes proportionally with the change of *w*, *b*, while the physical interval is fixed. When ‖*w*‖=1, the function interval is equal to the physical interval. The final optimization we need to complete is to select the classification plane that can maximize the minimum physical interval, as shown in

(5) $$\begin{array}{c} \underset{r,w,b}{\arg\max}\frac{\overset{\wedge }{y}}{w},\\ s.t.y_{n}\left(w^{T}x_{n}+b\right)\geq \overset{\wedge }{y}. \end{array}$$

In the formula, *s*.*t*. is abbreviated as constraint condition, where *n*=1,…, *N*.

The direct operation here will be very complex. We set the function interval of the sample closest to the classification interface to 1 by using the characteristic that the function interval changes in proportion to the change of *w*, *b* without affecting the physical interval. Then, we transform the original problem into a quadratic programming problem that is easier to solve:

(6) $$\begin{array}{c} \underset{w,b}{\arg\min}\frac{1}{2}w^{2},\\ s.t.y_{n}\left(w^{T}x_{n}+b\right)\geq 1, \end{array}$$

where *n*=1,…*N*.

To solve such problems, we usually combine the constraints and optimization problems into one formula through Lagrange factor. The Lagrange equation obtained is as follows:

(7) $$\begin{array}{c} L\left(w,b,a\right)=\frac{1}{2}w^{2}-\sum_{n=1}^{N}a_{n}\left\{y_{n}\left(w^{T}x_{n}+b\right)-1\right\}. \end{array}$$

Pay attention to the order of solution here, which is still to get the minimum physical interval according to *w*, *b* first, and finally to maximize the minimum physical interval. First, we find the partial derivative of Lagrange equation to *w*, *b* and make it equal to 0. Get the following two equations:

(8) $$\begin{array}{c} w=\sum_{n=1}^{N}a_{n}y_{n}x_{n},\\ \sum_{n=1}^{N}a_{n}y_{n}=0. \end{array}$$

After the above two equations are introduced, we get the duality problem of maximizing the physical interval. This dual problem only contains *a*, and after solving *a*, we can get *w*^*∗*^, *b*^*∗*^ by bringing it into the formula. The optimal interface is *w*^*∗T*^*x*+*b*^*∗*^=0.

(9) $$\begin{array}{c} \overset{\wedge }{L}\left(a\right)=L\left(w,b,a\right),\\ =\sum_{n=1}^{N}a_{n}-\frac{1}{2}\sum_{n=1}^{N}\sum_{m=1}^{N}a_{n}a_{m}y_{n}y_{m}x_{n}^{T}x_{m},\\ s.t.a_{n}\geq 0,\\ \sum_{n=1}^{N}a_{n}y_{n}=0. \end{array}$$

Type middle *n*=1,…*N*.

Finally, the 3D data acquired by using motion capture technology needs to be presented on the computer in a concrete model, and animation is generated for teaching and playing. Students can compare the learned dance movements with the teacher's standard movements by segments through the motion capture system, which can quickly find out the shortcomings and facilitate local correction.

## 4. Design of Recognition Model of Tumbling Posture in Classical Dance

### 4.1. Tumbling Posture Recognition of Classical Dance Based on Motion Capture Technology

The data acquisition in the tumbling posture process of classical dance is done using motion capture technology, and the skeleton motion route of the human body is extracted, followed by posture discrimination using the feature vector matching method to create the tumbling posture model of classical dance. The different postures of the human body are divided into two categories: static posture and dynamic posture; the recognition process of static action and dynamic action is carried out in the second level, respectively. The disadvantage of this structure is that it has a problem with error transmission, which means that misclassification samples from the first level will flow into the second level, resulting in a second-level classification error. The key to solving this problem is whether the system's design fully considers the inherent differences between static and dynamic posture, as well as the relative ease with which they can be distinguished. It is possible to interpret and classify multiple sensors at the same time. The results show that the first-grade classification error can be largely ignored, effectively suppressing the error propagation problem. Install 20 data identification points on each part of the dance trainer's body; then start the high-speed 3D data dynamic capture system while remaining well within the preset space range. The controller recognizes that the trainer has completed all of the preprogrammed basic movements. The dynamic capture system will track the dance movements and match them to the model in this process. The real-time acquisition of human action is completed when the computer successfully identifies and enters 20 data acquisition points into the system.

Based on the application of motion capture technology to the identification of the tumbling posture content of classical dance, various postures of human body are divided into two categories: one is static posture, and the other is dynamic posture. In the second level, the recognition process of static action and dynamic action is carried out respectively. The writhing gesture recognition form of classical dance based on motion capture technology is the intersection of computer science, educational technology, and educational psychology. By absorbing and learning from new theories, technologies and methods in other fields, the disadvantages of traditional recognition mode can be solved. The virtual display platform collects all kinds of dance materials, performs by actors, collects data through motion capture devices, and converts them into data recognizable by 3D animation software, and finally displays the dance content perfectly through the virtual display engine. After the motion capture system is successfully matched, the data of human motion posture is recorded, and the natural characteristics of human motion from different perspectives can be analyzed by the system software. In this paper, the motion model database uses key joint points to mark the movement changes of human body. At present, the connection between key points is mainly rigid connection, which can ensure the stability of dance posture. By comparing the dance movements with the teacher's standard movements in sections through the motion capture system, the shortcomings can be quickly found out, which is convenient for local correction. Motion capture technology is used to assist the teaching and research of dance.

### 4.2. Experimental Results and Analysis

In this experiment, taking the left arm movement of the dance trainer as an example, taking the left arm characteristic plane *p*_1_ as the basic calculation plane, three discriminant parameters {Sim(*V*_1_, *V*_stand_), Corr(*θ*_1_), Corr(*θ*_8_)} can be obtained, respectively, and the overall motion posture of the left arm can be determined by the above three parameters. Experiments show that the calculation error is effectively reduced, and the results are shown in Table 1.

After completing all teaching hours, the learning situation of the two groups of students is verified through assessment. The college dance teacher scores the range, strength, consistency, and technical standardization of aerobics actions of the two groups of students. The results are determined by SPSS19.0 analysis. The test results are shown in Table 2.

*p* represents the significance of the experimental effect, and *p* < 0.04 is generally the most significant. According to the experimental results, the students who learn by motion capture have a better grasp of dance movements than those who learn by routine.

This experiment was completed on a PC with Core (TM) i5-34703.2 GHz CPU and 5 GB memory, and MATLAB was used as the development environment. The created motion database contains 20 sets of dance action segments, each of which has about 1,300 frames. The subjects are randomly selected college students, and all subjects have dance foundation. Three experiments were carried out respectively, and the difference of left arm movement posture was compared. From Figures 3–5, the difference between the movement to be measured and the standard movement was clearly seen.

Through the comparison and verification of the experimental results in Figures 3–5, using the feature plane similarity matching method to analyze the motion posture can clearly and efficiently detect the differences and standards between moving objects and has high robustness, which lays a foundation for the scientific training of dance. Coordination is the basic quality of a dancer. The teaching of turning over covers the correct turning of the waist, the orientation training of hand posture, and the joint cooperation of crotch, leg, knee, foot, and step below the waist. It is a great test and exercise for the cultivation of coordination. If the body, especially turning over, is difficult to complete without coordination; even if it is completed, it will lack the corresponding beauty. Therefore, the coordination of turnover movement training dancers is a key point. Physical training can be divided into three stages: initial stage, middle stage, and later stage.

In this experiment, the peak frequency points in the tumbling posture of classical dance, such as basic turning, step-by-step turning, and step-by-step turning, were compared in two experiments. The experimental results are shown in Figures 6 and 7.

From Figures 6to 7, it can be seen that this feature shows a high degree of discrimination in the three categories of classical dance tumbling posture. At the 8th frame of the sample, the average frequency of step turn is 0.9, which is higher than the average rating of basic turn of 0.75 and that of point turn of 0.5. Therefore, it can be concluded that stepping over is an effective feature, except for some points with loud noise, which is generally stable. In the environment of motion capture equipment, students may have some adaptability problems, which are relatively restrained. However, students can make greater progress by simulating the posture of learning dance training and constantly revising their own learning process, especially in the standardization of dance movements, and students can realize their own shortcomings faster.

## 5. Conclusions

The motion capture system-based tumbling posture recognition of classical dance will not only play an important role in the protection of national dance, but also in the long-term development of national dance. The display of dances from various cultures can help with dance research, learning, development, and application. This paper examines human motion posture using the real-time characteristics of motion capture technology, proposes a tumbling posture recognition model for classical dance based on motion capture technology, examines the characteristics of human motion posture, examines the development prospects and research significance of using motion capture technology in classical dance, and provides an effective theoretical basis for scientific training. The range, strength, consistency, and technical standardization of aerobics actions of the two groups of students were scored by the dance teacher. The average frequency of step somersault is 0.9, which is higher than 0.75 of the average evaluation rate of basic somersault and 0.5 of point somersault, according to SPSS19.0 analysis. In addition to the large noise, it can be concluded that the overall turning point is effective. The motion capture technology proposed in this paper can recognize basic classical dance tumbling postures with high precision. The system's ability to achieve higher-precision recognition of more types of posture on this basis is critical. Dance teaching and research benefit from the use of motion capture technology. The captured specific three-dimensional motion data is transformed into digital abstract motion, the three-dimensional human body motion posture database is established, and the teaching animation video is generated, which helps to optimize the traditional dance learning form, according to the characteristics of real-time tracking, detection, and recording of motion capture technology. The importance of improving educational quality cannot be overstated.

## Figures and Tables

**Figure 1:** Dance posture flowchart of motion capture technology.

**Figure 2:** Basic skeleton structure of human body.

**Figure 3:** Difference of left arm movement direction.

**Figure 4:** Difference of included angle motion of left arm joint.

**Figure 5:** Angle difference between left arm and trunk.

**Figure 6:** Comparison chart of multisample peak frequency points.

**Figure 7:** Comparison chart of multisample peak frequency points.

**Table 1:** Relevant parameters of left arm action attitude.

Experimental object	Sim(*V*_1_, *V*_stand_)	*Corr*(*θ*_1_)	*Corr*(*θ*_8_)
Standard object	0.6847	0.9758	1.0124
Object to be tested	0.7125	0.8314	0.9847

**Table 2:** Comparison of experimental results.

Group	Movement range	Strength of action	Action coherence	Action standardization
General group	83.3 ± 6.5	79.7 ± 7.3	81.3 ± 7.8	78.5 ± 6.4
Experimental group	81.4 ± 6.8	81.7 ± 5.2	83.2 ± 3.3	82.3 ± 4.3
Significant *p*	0.032	0.027	0.024	0.041

## Data Availability

The data used to support the findings of this study are available from the corresponding author upon request.
